This article has been retracted.

# Factors affecting awareness of emergency contraception among college students in Kathmandu, Nepal

**DOI:** 10.1186/1472-6874-9-27

**Published:** 2009-09-17

**Authors:** Ramesh Adhikari

**Affiliations:** 1 Geography and Population Department, Mahendra Ratna Campus, Tribhuvan University, Kathmandu, Nepal; 2 Institute for Population and Social Research, Mahidol University, Salaya, Thailand

## Abstract

**Background:**

In Nepal, Emergency Contraception (EC) could play a critical role in reducing unintended pregnancies, but very few people aware about it. This paper aims to investigate the level of awareness and factors influencing awareness of EC among college students.

**Methods:**

A cross-sectional study was carried out in April-May 2006. Structured self-administered questionnaires were administered to 1,137 college students (573 males and 564 females) in Kathmandu valley. The association between awareness of EC and the explanatory variables were first assessed in bivariate analysis using the Chi-square test. The associations were further explored using a multivariate logistic analysis.

**Results:**

Only about two-thirds of college students (68%) had ever heard about EC. Bivariate analysis shows that males were more aware (72%) of EC than were females (64%). Similarly, the awareness level was significantly higher among younger, unmarried youth who were from outside Kathmandu Valley, who lived with friends, and who had received reproductive health (RH) education in school/college. The study also found that students' sex, permanent place of residence (district), and RH education are significant predictors of awareness of EC. Males are 1.5 times more likely to be aware of EC compared to females. Furthermore, students who lived in Kathmandu Valley were 41% less likely to be aware of EC than were students from outside Kathmandu Valley. On the other hand, those students who received RH education in school/college were almost nine times more likely to be aware of EC compared to those who did not receive such education.

**Conclusion:**

Awareness of the EC is low among college students in Nepal. Health education initiatives should target students as they are more likely to be sexually active. There is a need to further educate students about EC which can help to reduce unintended pregnancies, many of which result in unsafe abortion and take a large toll on women's health.

## Background

Emergency contraception (EC) is contraception administered after unprotected intercourse. EC is the only method women can use to prevent pregnancy after they have had unprotected sexual intercourse, have experienced a contraceptive failure, have remembered too late that they have forgotten to take their birth control pills, or have been forced to have sex against their will. EC is sometimes referred to as "morning-after" or "post-coital" contraception. EC is intend for occasional or emergency use only and not as a regular means of contraception. Formerly, EC was thought to be effective only within 72 hours, but recent studies have confirmed it is effective for up to 120 hours [1,2]. EC methods include taking special doses of ordinary birth control pills as well as inserting an intrauterine device (IUD). Depending on the method used, EC can reduce women's risk of becoming pregnant from a single act of intercourse by between 75 and 99 percent [3].

Each year, about 210 million women around the world become pregnant [4]. Among them, about 75 million pregnancies (36%) are unplanned and/or unwanted [5]. Unplanned/unwanted pregnancy is one of the leading causes of maternal mortality and morbidity in South Asia. Reasons for such huge numbers of unintended pregnancies in South Asia include a low rate of contraceptive use, method failure, and high unmet need for contraceptives. Each year worldwide, more than 20 million women experience ill health as a result of pregnancy [6]. It is estimated that between 8 and 30 million pregnancies each year result from contraceptive failure either due to inconsistent or incorrect use of contraceptive methods or failure of the method itself [7]. Research studies conducted in the USA have reported that higher rates of unintended pregnancy occur among college-age women, with 60% of pregnancies among 20-24 years old being unintended. The percentage of unintended pregnancy is even higher among 18-19-year-old females (79%) [8].

In Nepal, the data suggest that more than a third (35%) of all pregnancies [9] and 41% of the current pregnancy among currently pregnant women are unintended [10]. The prevalence of premarital sex has been reported as 39% among college males and 12% among college females [11]. A considerable proportion of both males (10%) and females (22%) reported that their first sexual intercourse happened without their consent. These students are at the greatest risk of unintended pregnancy. A study has also found that a large proportion of college students who were studying in Kathmandu (43% of males and 55% of females) did not use a condom during their first sexual intercourse [12].

Research on the awareness of EC among college students may help to inform policy makers and education planners in Nepal. Unfortunately, no research has been conducted in this area among the students in the country. The aim of our study is to investigate awareness levels and factors influencing awareness of EC among college students. We hope this study will provide baseline data to assist policy makers and education planners in developing appropriate evidence-based strategies and curricula in school/college to prevent unintended pregnancy and unsafe abortion.

## Methods

The institutional review board of the University Grant Commission (UGC), Nepal approved this study. The data used in this paper come from a cross-sectional survey on "Attitude and behavior towards pre-marital sex among college students of Kathmandu, Nepal" carried out in 2006.

A two-stage systematic random sampling technique was applied, the first stage of which included random selection of 12 colleges in Kathmandu. In order to select these 12 colleges, a list of all the private and public colleges affiliated with Tribhuvan University and located in Kathmandu Valley was obtained from the office of the Vice Chancellor in Kathmandu. This list included colleges which provide intermediate (commonly known as Grade 11 & 12), undergraduate, and graduate degrees. In the second stage, two classes were selected randomly from each sampled college. The number of students in a class ranged from 40 to 60. Since all the colleges were co-educational, all males and females students present on the day of the interview in the sampled classes were requested to participate in the study. Females and males students were interviewed separately in different classrooms. A self-administrated structured questionnaire in the Nepali language was used to obtain information from the students. The questionnaires were pre-tested among college students in a non-selected college and later refined as required. Almost all students in selected classes were present on the day of interview. None of the approached students refused to participate in the study. With regard to awareness of EC, the survey assessed awareness by asking the question, "Have you ever heard about emergency contraception?" [See additional file 1]. A total of 1,137 college students (573 males and 564 females) in Kathmandu Valley were interviewed.

Verbal informed consent was obtained from the participants before they were enrolled in the study. The consent form was written in the local language stating the study's objectives, nature of participant's involvement, risk and benefits, and confidentiality of the data. Students were requested to read the consent form carefully. They were given clear options on voluntary participation. It was also made clear that they could refuse to answer any questions and terminate the interview when they desired. Confidentiality of information was ensured by removing personal identifiers from the completed questionnaires. The names of sampled colleges are not made public and thus it is not possible for anyone outside the research team to trace reported incidents of sexual behavior to respondents. Respondents are thus protected against any possible adverse repercussions from participating in the study.

All completed questionnaires were entered into a database immediately after being manually coded and validated. Data entry and validity checks were performed for all the questionnaires by using the software program dBase IV. The cleaned and validated data was transferred into the SPSS 11.5 program for further processing and analysis.

Both bivariate and multivariate techniques were applied to identify the factors associated with the likelihood of being aware of EC. The Chi-square test was used to test the association. The variables that were significant in the bivariate analysis were reexamined in the multivariate analysis (binary logistic regression) in order to identify the significant predictors after controlling other variables.

## Results

A large majority of the respondents (85% males and 92% females) were in the youth category (15-24 years). An overwhelming majority of the students (88% of males and 83% of females) were unmarried, and 86% (91% of males and 80% of females) were from outside Kathmandu valley. Students covered in this study were from 67 districts out of 75 districts of the country. A majority of the males (59%) and about a quarter of the females (23%) lived either with friends or alone in Kathmandu. More than half of both males and females were currently pursuing their undergraduate degree. A large majority of the students (93% of the females and 91% of the males) had received education related to reproductive health in their respective schools/colleges (table not shown).

Overall, only about two-thirds of the college students (68%) had heard about EC. Table 1 shows a clear association between awareness of EC and other background variables such as sex and age of the students, level of education, marital status, permanent place of residence, types of current accommodation, and RH education in school/college. For example, male students were more aware (72%) of EC than were female students (64%). Similarly, a higher proportion of younger students aged 15-19 (73%) than the older students (66%) were aware of EC. Unexpectedly, a higher percentage of students (74%) who had an undergraduate level of education had heard of EC compared to those who had graduate or post graduate education (66%). Regarding marital status, unmarried students were more aware of EC than married students. Similarly, the awareness level was significantly higher among those who were from outside Kathmandu Valley, who lived either alone or with friends, and who had received reproductive health education in school/college. For instance, more than two-thirds of students (70%) who were from outside Kathmandu Valley while less than three-fifths (57%) of those who lived in Katmandu Valley were aware of EC. Likewise, those students who were living with their family members were less aware (66%) of EC than those who were living either alone or with friends (72%). A far higher proportion of the respondents who had received RH education in school/college (72%) had heard about EC than those who had not received RH education (24%) (Table 1).

**Table 1:** Awareness about Emergency Contraception by background characteristics

**Background characteristics**	**Awareness of EC**		**Number**	**χ^2^**
			
	**Yes**	**No**		
**Sex of the respondents**				P < 0.01
Females	64.2	35.8	564	
Males	72.3	27.7	573	

**Age group**				P < 0.05
15-19	72.5	27.5	418	
20 and above	65.8	34.2	719	

**Marital Status**				P < 0.05
Married	61.8	38.2	165	
Unmarried	69.3	30.7	972	

**Level of education**				P < 0.05
Intermediate	74.3	25.7	272	
Bachelors degree	66.3	33.7	629	
Masters degree	66.5	33.5	236	

**Permanent place of residence**				P < 0.01
Outside Kathmandu Valley	70.1	29.9	973	
Kathmandu Valley	57.3	42.7	164	

**Type of current accommodation**				P < 0.05
With family members	65.9	34.1	665	
Without family members	71.6	28.4	472	

**Received RH education in school/College**				P < 0.001
No	23.7	76.3	93	
Yes	72.2	27.8	1044	

**Total**	**68.2**	**31.8**	**1137**	**100.0**

**Table 2:** Odd Ratio (OR) and 95% Confidence Interval (CI) for having awareness about emergency contraception among college students

**Selected predictors**	**OR**	**95% CI**
**Sex of the respondents**		
Females (ref.)	1.00	
Males	1.50**	1.12-2.01

**Age group**		
15-19 (ref.)	1.00	
20 and above	0.83	0.58-1.19

**Level of education**		
Intermediate (ref.)	1.00	
Bachelors degree	0.85	0.57-1.26
Masters degree	0.89	0.53-1.47

**Marital Status**		
Married (ref.)	1.00	
Unmarried	1.19	0.82-1.72

**Permanent place of residence**		
Outside Kathmandu Valley (ref.)	1.00	
Kathmandu Valley	0.59**	0.41-.86

**Type of current accommodation**		
With family members (ref.)	1.00	
Without family members	0.96	0.71-1.31

**Received RH education in school/College**		
No (ref.)	1.00	
Yes	8.92***	5.38-14.78

**-2 Log likelihood**	**1309.4**	

**Cox & Snell R Square**	**0.094**	

Note ** Significant at P < 0.01, ***P < 0.001, ref = reference category

These observed associations in bivariate analysis were reassessed by logistic regression to identify adjusted association with the probability of being aware of EC. The results are presented in Table 2. As can be seen from the table, variables such as sex of the students, permanent place of residence (district), and RH education are significant predictors of awareness of EC after controlling for other variables. Males are 1.5 times more likely than females to be aware of EC. Similarly, students who lived in Kathmandu Valley were 41% (OR = 0.59, 95% CI = 0.41-0.86) less likely to be aware of EC than students from outside Kathmandu Valley. Likewise, those students who received RH education in school/college were almost 9 times more likely to be aware of EC compared with those who did not receive such education (Table 2).

## Discussion

The study looked at the awareness level and factors influencing awareness of EC among college students. Research shows that most college students had experienced unprotected sex and unintended pregnancy [8]. In such cases, EC could play a critical role in reducing unintended pregnancies. The awareness of EC among college students in Kathmandu is 66%, which is higher than the level found among university students in Kenya (39%) [13], Ghana (43%) [14] and Cameroon (63%) [15] On the other hand, it was very low compared to the university students, for example, in the USA (94%) [16] and Jamaica (84%) [17].

Although EC is not recommended as a routine family planning method, it is a very useful method after unprotected sexual intercourse to reduce the chance of unplanned or unwanted pregnancies. EC is an effective means of preventing unwanted pregnancies, but unfortunately the large numbers of college-going students are unaware of it. Analysis shows that male students were more likely to be aware of EC than were female students. It could be due to the fact that more males are living with their friends. The other reason could be that males are more open to talking with friends or seniors about issues of sex and sexuality than are females. Similarly, those respondents whose permanent place of residence is outside of Kathmandu were more likely to be aware of EC than were those whose permanent residence is in Kathmandu Valley. It was also found that almost all of the students whose permanent place of residence is Kathmandu were living with their family. This could cause them to be reluctant to talk about family planning methods or sex-related issues with their family members. The other reason might be that the students who live with friends are better informed by their peer groups.

In Nepal, students are taught subjects touching on health and population in school, including basic information on fertility, mortality, human reproductive organs, menstruation, and sexually transmitted infections including HIV/AIDS. Although the school or college health curriculum does not include EC, those students who had received RH education in school/college were more likely to be aware of EC than were those who had not. This may be because teachers who teach RH usually teach about risky sexual behavior, including the prevention of unwanted or unplanned pregnancies. Similarly these teachers usually teach the students about the emerging issues in reproductive health.

## Conclusion

Awareness about EC among college level students is low. Health education initiatives should target such students as they are more likely to be sexually active. There is a need to educate students about EC, which can help to reduce unintended pregnancies, many of which result in unsafe abortion and take a large toll on women's health. Education about EC at college levels could benefit even out-of-college youth, because their friends often are students.

## Competing interests

The author declares that they have no competing interests.

## Authors' contributions

RA, Lecturer of Mahendra Ratna Campus, Kathmandu, conceived and designed the study. He carried out the data collection, conducted data analysis and interpretation of the data.

## Pre-publication history

The pre-publication history for this paper can be accessed here:



## Supplementary Material

Additional file 1 **Questionnaire on the study entitled "Survey on Attitude and Behavior towards premarital sex among college students of Kathmandu Valley"**. The questionnaire includes various aspects of information regarding premarital sex, risky sexual behavior, HIV, emergency contraception etc. Click here for file
